This article has been retracted.

# Design and Innovation of Piano Impromptu Accompaniment for College Music Performance Majors under the Information Environment

**DOI:** 10.1155/2022/5245256

**Published:** 2022-07-08

**Authors:** Yanling Wang

**Affiliations:** Liaocheng University Dongchang College, Liaocheng, China

## Abstract

The development of information technology has a profound impact on the development of education. The integration of information technology into the teaching of professional courses has changed not only teaching methods and means, but more importantly, the teaching philosophy, teaching organization, and teaching evaluation are supported by information technology. Changes and progress have also been made. Piano improvisational accompaniment is an indispensable and important course in the teaching of music majors in colleges and universities. Relying on the information-based teaching environment and means, systematically designing piano impromptu accompaniment teaching for music performance majors to improve the effectiveness of teaching is a new exploration in the education and teaching reform of the current higher vocational music performance talent training courses. This study analyzes and studies the problems existing in the current teaching of piano improvisation accompaniment in colleges and universities and proposes the feasible strategies of piano improvisation accompaniment teaching in a targeted manner, to provide reference and guidance for the majority of educators.

## 1. Introduction

The “Opinions of the Ministry of Education on Accelerating the Development of Vocational Education Informatization” put forward that with the advancement of science and technology, to better conduct research on composition and piano accompaniment performance and teaching in the information age, it is necessary to change the relatively backward traditional teaching mode [1]. Because the traditional piano music teaching mode is mainly theoretical knowledge teaching and piano playing teaching, the long-term use of this teaching mode will not only affect students “learning enthusiasm, but also easy to shackle students” musical thinking and literacy, which is not conducive to its long-term learning and development.

It is a comprehensive professional direction of horizontal development that breaks through the boundaries of the original disciplines, including aesthetics, pedagogy, psychology, musicology, piano performance teaching, and educational methodology [2–4]. Piano accompaniment is an extremely complex and colorful art, it is an important part of the piano art, its appearance and development make the piano art become more brilliant and brilliant, especially in its accompaniment. It has mainly polyacoustic, polyphonic, symphonic, and harmonic characteristics.

In particular, the lack of relevant research on teaching reform has made the art of piano accompaniment largely stuck in the outdated, single-indoctrination traditional teaching method, the curriculum setting emphasizes technology over cooperation, the professional characteristics are not prominent, and the training objectives and teaching methods are inconsistent. Today, with the rapid development of information environment, artificial intelligence has been applied in all walks of life. In the deepening reform of piano teaching, we urgently need to build a modern teaching environment, build a big data platform for piano performance through information collection equipment, and use artificial intelligence technology to instantly evaluate and feedback the effect of students' piano performance as shown in Figure 1. Teachers and teaching assistants can provide one-to-one guidance and help according to the students' performance situation and requests, to improve the level and teaching efficiency of the piano impromptu accompaniment in the music performance major.

In addition to the problems existing in piano accompaniment art teaching, we also need to deal with the relationship between theory and practice. We need to face the problems existing in the teaching of piano accompaniment, deal with the relationship between theory and practice, break through the previous model, and enhance the operability of theory to guide practice [5, 6]. This study analyzes and studies the problems existing in the current piano impromptu accompaniment teaching in colleges and universities and puts forward the feasibility strategy of piano impromptu accompaniment teaching, to provide reference and guidance for the majority of piano accompaniment art educators.

## 2. An Overview of the Development of Piano Accompaniment

### 2.1. The Development Process of Foreign Piano Accompaniment Art

The piano has polyphony, harmony, polyphony, and symphony. The characteristics that other instruments do not have determine that the piano can become an accompaniment instrument that blends with human voices and other instruments. It has been more than 30 years since 1980 when the piano improvisation accompaniment class was officially included in the university curriculum.

The cooperation between piano and vocal music first appeared in the Baroque period. The accompaniment of this period used the form of continuo bass and mostly used the textured form of arpeggios and cylindrical chords. In daily opera rehearsals and small concerts, it is replaced by piano accompaniment. The band has become an inevitable choice for vocal accompaniment [7]. In the classical period, the accompaniment style of the piano was mainly based on the melody of the human voice, and the accompaniment parts were used as a foil. The structure was simple, the tone was uniform, and the sentences were clear. Entering the period of Romanticism, the appearance of Schubert's art songs raised the status of piano accompaniment to an unprecedented height. During the Romantic period, Schumann, Mendelssohn, Brahms, and Rachmaninoff created numerous piano duets and quartets, and their classic works are still active in the performance stage of chamber music [8]. During this period, the piano accompaniment used a large number of modulations and dissonances, the harmony colors became richer, the texture forms became more diverse, and the dynamic changes became more eclectic. With the development of the economy and the continuous heating up of the piano career, the piano improvisation accompaniment course has attracted the general attention of teachers and students, and the piano improvisation accompaniment course has also become a compulsory course for music education majors in major music colleges and universities, and the theoretical research results related to it have also emerged.

### 2.2. The Opening of Piano Accompaniment in Foreign Music Schools

In the postgraduate entrance examination, piano accompaniment is a compulsory test and a compulsory course in the future. Germany and Austria are generally regarded as sacred places of classical music with profound musical culture, and major music schools have established the piano accompaniment art direction at the postgraduate level, and the professional structure, curriculum, and teaching system are very complete. The old concept that piano accompaniment practitioners are regarded as “second-class citizens” no longer exists. In classroom and stage practice, teachers and students from different majors understand and respect each other, establish a good cooperative relationship, and gradually realize that Piano accompaniment is a very good career direction.

### 2.3. The Experience and Enlightenment of Foreign Piano Accompaniment Teaching Practice

The talent training objectives, teaching concepts, curriculum setting, teaching methods, and examination methods are closely combined. As shown in Figure 2, the talent training objectives, teaching concepts, curriculum settings, teaching methods, and examination methods in the direction of foreign piano accompaniment are closely integrated. The curriculum settings of foreign music schools are closely integrated with their training objectives, and all curriculum settings can reflect their training objectives [9]. In terms of training objectives and curriculum settings, the foreign piano accompaniment art major aims to cultivate “practical” cooperative talents, and the courses are mostly practical courses. Foreign music academies pay attention to the traditional inheritance of music culture and offer courses such as “clave” and “ancient music” with profound traditional cultural heritage. Some colleges also offer vocal singing courses, which require students to understand the methods of vocal singing and lay a good foundation for cooperation with vocal singers, such as the Cologne Conservatory of Music in Germany; some colleges set different course modules, including compulsory and elective, and after the completion of the course of each module, a certificate of completion will be given by examination, and students will also receive corresponding credits. The school provides public classes and “one-to-one” small classes with multiple teaching and research offices, and teachers teach in course examinations and concerts. Result assessment and evaluation: teachers often bring the latest research results into the classroom to give full play to the autonomy of students. Instead of “teacher-centered,” they focus on the diversity of teaching and students' initiative and independence in learning. The examination and evaluation system is divided into entrance examination, school year examination, and graduation examination. This shows that foreign music schools have a clear goal of training talents in piano accompaniment art. In the academic year examination, foreign music schools have adopted different methods. In the graduation examination, foreign music schools usually require to hold a degree concert and write a degree thesis, and in these two links, foreign music schools pay more attention to concerts [10]. Through the experience and enlightenment of the abovementioned foreign piano accompaniment teaching practice, this article will address these problems, and we must take some countermeasures to improve the teaching of piano improvisational accompaniment, thereby improving students' improvisational accompaniment ability to promote the development of music education in colleges and universities.

## 3. Investigation and Analysis of the Current Situation of Piano Teaching Development in Performance Majors

According to the preliminary literature research, I learned the current situation of piano accompaniment in the performance field and selected all the schools majoring in piano performance to conduct a questionnaire survey on students majoring in piano performance, to understand and analyze the relevant situation of students majoring in piano performance.

### 3.1. Basic Situation

It can be seen from Table 1 that the descriptions of the training objectives of the three institutions are different, some are relatively clear, and some are not clear enough. The author checked the training objectives and curriculum schedule of the Central Conservatory of Music, China Conservatory of Music, and Wuhan Conservatory of Music. The curriculum settings of the three colleges can all focus on the training objectives, and the settings are relatively extensive, but they fail to reflect the attention and change in social needs. Nowadays, colleges and universities generally lack music aesthetics and courses combined with Chinese traditional music culture, and the proportion of cooperative practice is not high, which is not conducive to the cultivation of the basic quality and ability of piano accompaniment talents, and also affects the competitiveness of students after graduation.

Curriculum setting mainly refers to setting course categories, course types, course schedules, and hour allocation around the goal of talent training in colleges and universities and formulating specific course learning objectives, learning requirements, and learning content, which are mainly composed of course structure and course content. The training goal of piano accompaniment art under the concept of “work-centered” requires students to attach importance to professional performance skills, master a certain depth of music theory, and have considerable artistic aesthetic ability, as shown in Tables 2-3.

From Table 4, we can see the age of piano teachers. The number of teachers under the age of 35 is 1, accounting for 10% of the total number; the number of teachers between the ages of 36 and 50 is 6, accounting for 60% of the total number; and the number of teachers over 50 years old is 3, accounting for 30% of the total number. This reflects that the overall age distribution of piano teachers in the music department is between 36 and 50 years.

This survey is conducted on undergraduate and graduate students majoring in music performance. The number of surveyed is 19, the total number of questionnaires distributed is 19, the actual number of questionnaires returned is 13, and the number of valid questionnaires is 13, accounting for 10% of the total 68%. The number of first-year graduate students is 2, accounting for 15% of the surveyed population; the number of second-year graduate students is 1, accounting for 8% of the surveyed number; and the number of undergraduate first-year students is 1, accounting for the total surveyed. The number of students in the second year of undergraduates is 5, accounting for 23% of the total number of students surveyed; the number of students in the third year of undergraduate studies is 3, accounting for 38% of the total number of students surveyed; and the number of students in the fourth year of undergraduate studies is 1 person, accounting for 8% of the total number of respondents. The data results are summarized in Figure 3: according to the above analysis, the number of students majoring in music performance is polarized. The higher the grade and the lower the grade, the smaller the number of students, which reflects the small number of students majoring in music performance, and it is difficult to stick to it because of the high difficulty of the major.

## 4. The Teaching Reform Goal Orientation

The reform of piano accompaniment teaching is rooted in teaching practice, and its purpose is to reveal the inherent laws of cultivating multilevel and all-round development of piano accompaniment talents and art instructors. As an organic part of music teaching in colleges and universities, improvisational piano accompaniment is of great significance to improving students' musical ability and the development of music education in colleges and universities. My country's higher music colleges have not yet established a complete and mature education system, and there are many problems, such as short school time, weak foundation, backward training concepts, excessive teaching mode inertia, low degree of innovation, and little subjectivity for students to learn, the classroom practice is not cooperative, the teaching evaluation system is single, and so on. As shown in Figure 4, it reflects the urgent needs of the whole society for improving the teaching quality of piano accompaniment and cultivating new high-quality piano accompaniment workers and establishing the teaching reform goal of piano accompaniment art. It has important practical significance.

### 4.1. Clarify the Professional Functions of Piano Accompaniment and Cultivate Students' Quality Ability

The direction of piano playing is both closely related and different. What needs to be clarified in the teaching reform is that the cultivation of performance ability is the foundation, and the cultivation of accompaniment cooperation ability is the top priority of professional functions. After taking the job, students can clear the direction and goal when facing the actual teaching work and be able to target and take charge of themselves. Piano accompaniment is a measure to test the level of students' piano performance skills. Often when applying for a unit, it will be used as an important test item to judge the ability of students. Therefore, improving students' accompaniment ability is also a part of talent training [11]. To improve the ability of piano accompaniment, first of all, in daily learning, students should be required to practice more so as to be familiar with the scales and arpeggios. Secondly, in the piano teaching, the piano students majoring in music education and music performance can be assigned a normal score accompaniment to improve the students' own sight-reading ability. The piano accompaniment can also be used in the ensemble of ethnic musical instruments, fully integrating a Western imported product such as the piano into the ethnic music culture and using the 88 black and white keys of the piano to authentically play the charm of ethnic music, which makes this music. The charm of a variety of folk music sprinkles between each note [3].

The ability to play and sing by yourself is also a very important teaching content. In the actual piano teaching, teachers can increase the repertoires that students play and sing and can also use it as a part of the final examination, to improve the students' high attention to this skill. In practical teaching, teachers can also use simple Xinjiang minority children's songs as teaching repertoires. According to students' playing and singing, teachers can give correct guidance, so that students can deeply realize the mutual cooperation between playing and singing. In practice, play and sing separately first.

### 4.2. Optimizing the Course Structure Setting and Building a Systematic and Perfect Teaching Mode

The setting of course content is an organic composition of teaching methods, and the selection of teaching mode is an indispensable basic link in the teaching process, and there are an inherent correlation and unity between the two. The traditional teaching mode focuses on the specific guidance of piano literature and piano performance and lacks a scientific attitude and multidimensional analysis for the cooperation of accompaniment and other musical instruments (singing parts). Only by recognizing the essential characteristics of all aspects of the teaching system and making a dynamic analysis of teaching practice from multiple perspectives we can construct a set of systematic and perfect teaching theories and methods that play a theoretical guiding role in piano accompaniment teaching.

The cooperation and mutual assistance model refers to the mutual cooperation between teachers and students, and between students and students, as shown in Figure 5. This model can effectively enhance the emotional communication between teachers and students and between students, to achieve mutual respect and trust between teachers and students. The characteristics of this model are mutual respect, mutual trust, mutual cooperation, and shared responsibility among cooperative partners, which can generate positive emotions for teachers, students, and others in teaching and learning and form better interpersonal relationships. Conducive to the overall development of the discipline and the common growth of students, its advantages are as follows: stronger motivational synergy can be generated in a cooperative environment than in an individual, competitive learning environment; members of a cooperative group learn from each other, and each member can both play a greater role than acting alone; and interpersonal interactions in cooperative groups can complicate cognitive and social learning, providing more benefits for learning than independent learning performance-enhancing intellectual activities. Then, this model in the piano teaching process also emphasizes a kind of cooperation and cooperation.

### 4.3. Clearly Study the Practical Significance of Piano Accompaniment Teaching Reform for Performance Majors

The improvisational accompaniment of the piano can integrate the performance and creation of the music and has practical value that cannot be ignored. The teaching of piano improvisational accompaniment needs to be continuously improved and improved, and attention should be paid to the teaching of the basic skills of student accompaniment, guiding students to appreciate different styles of musical works, cultivating students' skillful improvisational accompaniment skills and analytical ability, playing ability, sound arrangement ability, etc., enriching students' musical expression and creativity, and comprehensively improving students' musical literacy. Studying the teaching reform of music performance piano accompaniment can improve the quality of teaching, shorten the training period, and provide a theoretical basis for teaching practice.

### 4.4. Reform of Teaching Methods

The improvisational accompaniment of the piano can integrate the performance and creation of the music and has practical value that cannot be ignored. The teaching of piano improvisational accompaniment needs to be continuously improved and improved, and attention should be paid to the teaching of the basic skills of student accompaniment, guiding students to appreciate different styles of musical works, cultivating students' skillful improvisational accompaniment skills and analytical ability, playing ability, sound arrangement ability, etc., enriching students' musical expression and creativity, and comprehensively improving students' musical literacy.

#### 4.4.1. Teaching Method Design of Practical Class

Practical class is an important bridge connecting classroom teaching and stage practice, and the purpose is to improve students' stage practice ability and collective cooperation awareness. The “one-to-one” individual teaching form enables teachers to give full play to their leading role and organize teaching according to the individual characteristics of each student, fully protecting, respecting, and shaping students' sensibility and comprehension of performance techniques and musical styles. In view of the characteristics that students in higher music colleges are adults, we need to establish a learner-centered, interactive multilateral teaching method that emphasizes learner participation. In the traditional teaching, the teacher's dominance is too strong, the learning situation under the teacher's guidance is overemphasized, and the students are already adults who can think and solve problems independently. A large number of psychological studies have shown that what adult students need most in the cognitive process is participation, and the best learning situation is cooperation and interaction [12–14]. In the teaching of practical courses in higher music colleges, teachers should change the teaching method of “teaching by heart” and mobilize students' awareness of active participation suggestions and solutions. The interactive and multilateral teaching method breaks through the traditional one-way activity theory. It emphasizes that teaching activities are a kind of multilateral activities and advocates multilateral activities between teachers and students, students, and teachers, so that teaching can be carried out in multiple interactions. A three-dimensional information exchange network is formed. Because students often come from different growth environments, cultural and regional differences enable them to bring many fresh teaching experiences to teaching, which greatly enriches teachers' teaching resources and promotes mutual learning in teaching.

While inheriting the essence of traditional teaching methods, we need to cultivate students' innovative thinking and form teaching methods that teach, inspire, and guide; that is, students design performance methods—students tell about the creative background, aesthetic ideas, musical forms, and styles of works—student performance, teacher-student discussion, student recreation, and stage practice. This teaching method fully respects students' individuality, mobilizes students' initiative and innovation, and encourages students to use various learning tools, think independently, draw inferences from one case, and reasonably construct their own knowledge system and performance style. The traditional teaching method of the accompaniment art small class often omits the partner, and the teacher and the students only teach the accompaniment part, ignoring the internal and external connection between the singing (the sound of the piano) and the piano accompaniment, and cannot form a tacit cooperation and joint research on the works [3]. The new collaborative teaching method should invite appropriate collaborators into the classroom according to the works played, and the purpose is to guide the collaboration between the students and the singer (player) and realize the perfect dialogue between the piano accompaniment and the singing (the sound of the piano) [8].

To arouse students' interest in learning and the motivation to create chamber music, we should implement “discussion-style” teaching in our teaching. According to the students' individual professional skills and the needs of the students, teachers will comment on the works and performance cooperation, discuss the style, skills, art history theory, etc., of the works, and pay attention to cultivating students' creative, practical, and thinking abilities. The innovations are as follows: (1) students can “designate teachers,” and the selected teachers can teach one-person or group-group courses according to their own theoretical and practical research, students' confusion, and needs [15]. (2) Collective music group teaching: a chamber orchestra is set, and music group activities are conducted once a month to provide students opportunities and platforms for practice. Teachers and students of relevant majors can freely display, communicate, and interact in depth, strengthen communication and collaboration, and relieve students' confusion and blind spots in their learning. Students can hold concerts, record CDs, participate in various competitions and social practice performances, and assist teachers in conducting research on related topics. Through theoretical study, practice, and performance training, it helps students to experience the artistic beauty of piano accompaniment art in a three-dimensional manner, cultivates a sense of teamwork with others, exercises on-the-spot psychological quality, stimulates enthusiasm for learning, and forms a “learning-practice-re-learning-re-practice concept.” College students need to improve their practical experience and accumulate cooperation experience to improve their adaptability to future work.

#### 4.4.2. Teaching Method Design of Theoretical Courses

For a long time, theoretical courses in our country have been dominated by a teaching method that can be called “indoctrination.” Its main manifestations are attaching importance to specialized knowledge and skills and emphasizing on the imitation or application of existing achievements; it lies in and precedes the teaching process, and once it is set, it runs through the entire curriculum and remains unchanged, and the educational purpose becomes trivial. This teaching method regards students as a container, and the whole process and purpose of teaching are all about how to effectively instill knowledge into this container, which leads to a one-sided understanding of the value and goals of the course, ignoring aesthetic experience and life experience, and attaching importance to music The teaching and training of knowledge and skills despise the performance and appreciation of music. The harm of indoctrination teaching method is that teachers and students aim to memorize knowledge points by rote, disregarding students as subjects with personality, life, and thinking [16].

The teaching of theoretical courses should focus on the communication between teachers and students while teaching knowledge. Teachers should teach with an equal attitude, listen to the voices of students, and treat students as friends rather than objects of conquest, suppression, and subjugation. The American psychologist Bruner actively advocates the “discovery method,” also known as the “problem method,” that is, to find problems, answer them, and try to solve them. The spirit of exploration is as important as artistic innovation. In the teaching process, it is not a process of telling students the given answer, but a process of jointly researching music knowledge through teachers' analysis, description, inspiration, questioning, demonstration, and doubt-solving [17].

## 5. Conclusion

With the gradual attention of the state to education, the content of quality education has been further implemented, and the students' piano improvisational accompaniment ability can directly show the overall level of students' piano learning. Piano improvisation is also an important goal of piano teaching in music majors in colleges and universities, which directly affects the comprehensive quality and artistic literacy of students. Today, in the profession of music education, the art of vocal music is closely related to the performance effect of piano improvisation, and it is also a skill that students must have. Although the teaching of piano improvisational accompaniment is of great significance in music education, there are still many problems in terms of the actual teaching situation in China, which in turn has a greater impact on the teaching effect. On the basis of analyzing the existing problems in today's piano improvisational accompaniment classroom teaching, this study explores the effective strategies of piano improvisational accompaniment classroom teaching, hoping to promote the overall development of music education in colleges and universities.

## Figures and Tables

**Figure 1:** Information-based piano teaching mode.

**Figure 2:** Dimension setting of foreign piano accompaniment art training.

**Figure 3:** Number of students.

**Figure 4:** Problems existing in higher music colleges in China.

**Figure 5:** Cooperation and mutual assistance mode between teachers and students.

**Table 1:** List of training objectives for graduate students in piano accompaniment art in three professional music schools in China.

Colleges	Training objectives
Central Conservatory of Music	Cultivate senior talents engaged in vocal piano accompaniment and vocal music teaching guidance
China Conservatory of Music	Cultivate “complex talents” demanded by society
Wuhan Conservatory of Music	Cultivate a good performance level and a profound theoretical foundation, and be able to undertake teaching and scientific research

**Table 2:** Traditional course structure diagram.

Course title	Function	Credits	Course nature	Semester and arrangement
Main course (piano performance)	Performance technique	8	Main courses/compulsory courses	1-2/academic year
Main course (accompaniment art)	Accompaniment technology	8	Main courses/compulsory courses	1-2/academic year
Language class (Italian)	Guidance function	2	Major required	1st year/on
Dissertation writing guidance course	Cultural cultivation	2	Major required	1st year/second
Vocal art history	Art cultivation	2	Major required	Year 2/I
Vocal literature research	Art cultivation	2	Major required	1st year/first
Classical music version studies	Art cultivation	2	Major electives	2nd year/first
Music performance course	Art cultivation	2	Major elective	Year 2/second
Non-musicology courses	Cultural cultivation	2	General elective	Year 2/second
Total credits		30		

**Table 3:** Curriculum structure under the concept of “work-centered.”

Course title	Features	Credits	Course nature	Semester and schedule
Main lesson (piano performance)	Playing technique	4	Main subjects/compulsory courses	1st/school year
Main lesson (accompaniment art)	Accompaniment technique	8	Main subjects/compulsory courses	1-2/academic year
Impromptu piano accompaniment	Ethnic/cooperative	2	Required for majors	Year 1/second
Chamber music	Play together	8	Required for majors	Years 1-2
Language lessons (Italian)	Guidance function	2	Required for majors	Year 1/upper
Thesis writing instruction	Artistic accomplishment	2	Required for majors	Year 2/first
History of Western vocal art	Artistic accomplishment	2	Professional elective	Year 1/upper
Language class (German)	Guidance function	2	Professional elective	Year 2/first
Transpose and transpose	Artistic accomplishment	2	Required for majors	Year 2/second
Opera art appreciation	Artistic accomplishment	2	Professional elective	Year 1/upper
Total reading	Artistic accomplishment	2	Required for majors	Year 1/second
Musical aesthetics	Aesthetic function	2	Professional elective	Year 1-2
Vocal literature research	Cultural accomplishment	2	Professional elective	Year 1/second
Non-music graduate electives	Cultural accomplishment	2	General elective	Year 1-2
Total credits		42		

**Table 4:** Teaching age of teachers.

Age	≤35	36–50	≥50
10 people	1 people	6 people	3 people

## Data Availability

The labeled data set used to support the findings of this study is available from the corresponding author upon request.
